The article "Investigation of the Clinical Efficacy of Acupuncture Combined with Traditional Chinese Medicine Fumigation in the Treatment of Rheumatoid Arthritis by Meta-Analysis" was retracted in 2023. Reasons: signs of a paper mill; suspected computer-generated content; unreliable results or conclusions; concerns about the data.

# Investigation of the Clinical Efficacy of Acupuncture Combined with Traditional Chinese Medicine Fumigation in the Treatment of Rheumatoid Arthritis by Meta-Analysis

**DOI:** 10.1155/2022/7998725

**Published:** 2022-08-20

**Authors:** Weijing Tao, Qian Zhang, Lijuan Wang

**Affiliations:** ^1^Geriatric Medicine Center, Department No. 2 of Acupuncture & Massage, Zhejiang Provincial People's Hospital (Affiliated People's Hospital, Hangzhou Medical College), Hangzhou 310024, China; ^2^Geriatric Medicine Center, Department of Geriatric Medicine, Zhejiang Provincial People's Hospital (Affiliated People's Hospital, Hangzhou Medical College), Hangzhou 310024, China; ^3^Center for General Practice Medicine, Department of Rheumatology and Immunology, Zhejiang Provincial People's Hospital (Affiliated People's Hospital, Hangzhou Medical College), Hangzhou 310014, China

## Abstract

In order to investigate the clinical efficacy of acupuncture combined with traditional Chinese medicine fumigation in the treatment of rheumatoid arthritis (RA) by meta-analysis, literature related to the treatment of rheumatoid arthritis by acupuncture combined with traditional Chinese medicine fumigation are searched in line with the research direction. Meta-analysis is conducted by RevMan 5.2 software. A total of 17 literature are included and the publication bias of the included literature is low. The experimental results show that acupuncture combined with traditional Chinese medicine fumigation can reduce the inflammatory response and clinical symptoms of RA patients, and the addition of acupuncture can improve the clinical efficacy, which has a certain feasibility of promotion.

## 1. Introduction

Rheumatoid arthritis (RA) is a chronic immune disease with a high incidence, which is characterized by irreversibility and a high disability rate. The disability rate of RA patients suffering from rheumatoid arthritis for 5 to 10 years is as high as 43.5% and the coverage of the onset age is wide. Morning stiffness, pain, and swelling are common clinical manifestations. The longer the disease lasts, the higher the disability rate [1, 2].

The early clinical manifestations of RA patients are not obvious, which often leads to delay of diagnosis and treatment and affects the prognosis of patients. At present, western medicine treatment mainly uses antirheumatism drugs, hormones, and other drugs to control the disease, but the effect fails to achieve the expected results, and patients with long-term drug tolerance are poor and prone to adverse reactions [3]. Therefore, it is of great significance to explore effective and safe treatment for RA. Currently, there is a lack of medical evidence for acupuncture and moxibustion combined with traditional Chinese medicine fumigation in the treatment of RA.

The article "Investigation of the Clinical Efficacy of Acupuncture Combined with Traditional Chinese Medicine Fumigation in the Treatment of Rheumatoid Arthritis by Meta-Analysis" was retracted in 2023. Reasons: signs of a paper mill; suspected computer-generated content; unreliable results or conclusions; concerns about the data.

The rest of this paper is organized as follows: Section 2 discusses related work.  Section 3 discusses the literature screening criteria and quality evaluation. The evidence for clinical diagnosis and treatment is discussed in Section 4.  Section 5 concludes the paper with summary and future research directions.

## 2. Related Work

In recent years, acupuncture and traditional Chinese medicine fumigation have achieved definite efficacy and high safety in the treatment of RA, whose efficacy and safety have been verified in a number of research reports [4].

From the perspective of Traditional Chinese medicine, rheumatoid arthritis belongs to the category of arthralgia. The main pathogenesis is that the body is affected by wind cold and damp heat, which eventually leads to the blockage of blood vessels, pain, numbness, acid swelling, deformation, swelling, and other symptoms of skin surface blood vessel cells. If the disease is not controlled in time, it will invade the liver, kidney, and other important organs. Therefore, timely and effective treatment for RA patients is of great significance to their life safety [5]. Traditional Chinese Medicine (TCM) fumigation can achieve the therapeutic objectives from the outside to the inside and from the inside to the outside in the clinical treatment of RA, and can effectively improve the patients' qi and blood imbalance and meridians occlusion [6]. Acupuncture is China's traditional medical technology to effectively improve joint function and clinical symptoms in patients with rheumatoid joint, acupuncture and other treatments [7].

Joint swelling, pain, and morning stiffness are the main indicators for the clinical diagnosis of RA patients, which have certain guiding significance for the clinical diagnosis and treatment of RA patients [8]. Acupuncture can play a good role in relaxing tendons and activating blood circulation, thus playing a significant analgesic and detumescent effect [9].

As autoimmune diseases, one of the more than rheumatoid arthritis associated with abnormal immune system and inflammation, by the liver synthesis and secretion of C-reactive protein (CRP) is a kind of acute reactive protein. Moreover, it is a good predictor of reflecting the inflammation, so changes by laboratory monitoring CRP level can effectively reflect the condition of patients with RA developments [10]. Traditional Chinese acupuncture relieves inflammation and further reduces the abnormal increase of CRP [11].

## 3. Literature Screening Criteria and Quality Evaluation

### 3.1. Literature Retrieval

Randomized controlled trials (RCT) are used as the literature retrieval type. The retrieval direction is the value of acupuncture combined with TCM fumigation in the treatment of RA. TCM fumigation, rheumatoid arthritis, C-reactive protein, clinical symptoms, inflammatory factors, therapeutic therapy, Chinese herbal fumigation, and rheumatoid arthritis, C-reactive protein, clinical symptoms, inflammatory factors, efficacy, and other keywords are searched within 7 years in domestic and foreign literature databases such as Wanfang Medicine, Chinese National Knowledge Infrastructure (CNKI), and PubMed. Based on acupuncture, meta-analysis is conducted by RevMan 5.2 software on the basis of selected literature.

The article "Investigation of the Clinical Efficacy of Acupuncture Combined with Traditional Chinese Medicine Fumigation in the Treatment of Rheumatoid Arthritis by Meta-Analysis" was retracted in 2023. Reasons: signs of a paper mill; suspected computer-generated content; unreliable results or conclusions; concerns about the data.

### 3.2. Literature Screening Criteria

Inclusion criteria contains the following information: (1) The study plan is to use TCM fumigation and TCM fumigation combined with acupuncture. (2) Nationality, age, gender, race, and other restrictions are not set for the screening of research objectives. (3) The rate of loss to follow-up during the follow-up is less than 20%. (4) There are relevant institutions to review and approve documents. (5) Publication time is less than or equal to 7 years. (6) The original data are complete and there is no operation error. (7) The outcome indexes include total clinical response rate, clinical symptoms, pain score, and any one or more of CRP.

Exclusion criteria contains the following information: (1) Insufficient literature such as repeated content and loose operation. (2) Animal experiments. (3) Irrelevant to the research topic.

Literature outcome indicators contain total clinical response rate, morning stiffness time, joint tenderness score, joint swelling score, pain score, and C-reactive protein.

### 3.3. Quality Evaluation

The modified Jadad score scale is used to evaluate the quality of randomized controlled studies. The total score of the scale ranges from 1 to 7, with ≤3 as low qualities and ≥4 as high qualities.

RevMan5.2 statistical software is used to analyze the study data, and the counting data is expressed as risk ratio (RR). Weighted mean difference is selected as analysis statistics. All effect sizes are expressed with 95% confidence interval (CI). The heterogeneity between the results of each study is tested by a Chi-square test. When the heterogeneity between studies is statistically significant *P* < 0.1, subgroup or sensitivity is used to analyze the source of this property. When the heterogeneity between studies meet the conditions of *P* > 0.1, the heterogeneity has no statistical significance, and the fixed effect model is used for meta-analysis. When the source of heterogeneity is not clear, the random effect model and descriptive analysis of obvious clinical and methodological heterogeneity are used in the analysis.

The article "Investigation of the Clinical Efficacy of Acupuncture Combined with Traditional Chinese Medicine Fumigation in the Treatment of Rheumatoid Arthritis by Meta-Analysis" was retracted in 2023. Reasons: signs of a paper mill; suspected computer-generated content; unreliable results or conclusions; concerns about the data.

## 4. Experimental Results

According to the restricted conditions, 300 literature are retrieved from Chinese and English contributing databases and 17 literature are included after screening according to the literature inclusion criteria, including 16 Chinese literature and 1 English literature.  Figure 1 shows the specific retrieval process [12]. A total of 7 included literature are of low quality and 10 are of high quality.

The basic characteristics and quality evaluation results of included literature are shown in Table 1. In Table 1, A represents total clinical effective rate, B represents reactive protein, C represents pain score of visual analog scale, D represents morning stiffness, E represents joint swelling, and F represents joint tenderness.

Figure 2 shows the overall literature publication bias. It is clearly evident from Figure 2 that there is no significant publication bias.

Figure 3 shows the publication bias of single literature. It is clearly evident from Figure 3 that there is no significant publication bias.

### 4.1. Meta-Analysis of the Efficacy of Acupuncture Combined with Chinese Herbal Fumigation in RA

A total of 15 literature are included. The heterogeneity test show that there is heterogeneity among literature (I^2^ = 55.0%, *P*=0.005) and a random effect model is used for analysis. The total clinical effective rate of the combined group is significantly higher than that of the Chinese herbal fumigation group. There are statistically significant differences between the combined studies (RR: 1.21, 95%, CI: (1.13, 1.31), *P* < 0.00001).  Figure 4 shows meta-analysis of therapeutic effects of acupuncture combined with Chinese herbal fumigation on RA. It is clearly evident from Figure 4 that acupuncture and moxibustion combined with Chinese herbal fumigation can improve the total clinical response rate of RA patients.

### 4.2. CRP Meta-analysis of Acupuncture Combined with Traditional Chinese Medicine Fumigation in RA

A total of 3 literature are included, and the heterogeneity test shows that there is heterogeneity among literature (I^2^ = 99.00%, *P* < 0.00001). The CRP level in the combination group is significantly lower than that in the traditional Chinese medicine fumigation group and the difference is statistically significant (RR: 5.01, 95% CI: (−5.99, −4.02), *P* < 0.00001).  Figure 5 displays the forest map of CRP meta-analysis of ACUPUNCTURE combined with Chinese herbal fumigation in RA treatment. It is clearly evident from Figure 5 that acupuncture combined with traditional Chinese medicine fumigation can reduce CRP level in RA patients.

The article "Investigation of the Clinical Efficacy of Acupuncture Combined with Traditional Chinese Medicine Fumigation in the Treatment of Rheumatoid Arthritis by Meta-Analysis" was retracted in 2023. Reasons: signs of a paper mill; suspected computer-generated content; unreliable results or conclusions; concerns about the data.

### 4.3. Meta-Analysis of Clinical Symptoms of RA Treated by Acupuncture Combined with Chinese Herbal Fumigation

A total of 10 literature are included and the heterogeneity test shows that there is heterogeneity among literature (I^2^ = 96.00%, *P* < 0.00001) and the VAS pain symptom score of the combined group is significantly lower than that of the traditional Chinese medicine fumigation group, and the difference is statistically significant (RR: −1.55, 95% CI: (−1.62, −1.47), *P* < 0.00001).  Figure 6 shows VAS score meta-analysis of acupuncture combined with Chinese herbal fumigation for RA. It is clearly evident from Figure 6 that acupuncture combined with traditional Chinese medicine fumigation can alleviate the VAS pain symptoms of RA patients.

A total of 8 literature are included, and the heterogeneity test shows that there is heterogeneity among literature (I^2^ = 87.00%, *P* < 0.00001). The time of morning stiffness in the combined group is significantly shorter than that in the traditional Chinese medicine fumigation group and the difference is statistically significant (RR: −13.73, 95% CI: (−14.97, −12.49), *P* < 0.00001).  Figure 7 shows meta-analysis of morning stiffness time of RA treated by acupuncture combined with Chinese herbal fumigation. It is clearly evident from Figure 7 that acupuncture combined with traditional Chinese medicine fumigation can shorten the time of morning stiffness in RA patients.

A total of 8 literature are included, and the heterogeneity test shows that there is heterogeneity among literature (I^2^ = 98.00%, *P* < 0.00001). The joint swelling symptom score in the combined group is significantly lower than that in the traditional Chinese medicine fumigation group and the difference is statistically significant (RR: −0.42, 95% CI: (−0.47, −0.36), *P* < 0.00001).  Figure 8 shows meta-analysis of the joint swelling symptom score of acupuncture combined with Chinese herbal fumigation in RA. It is clearly evident from Figure 8 that acupuncture combined with traditional Chinese medicine fumigation can reduce the symptoms of joint swelling in RA patients.

A total of 6 literature are included, and the heterogeneity test shows that there is heterogeneity among literature (I^2^ = 96.00%, *P* < 0.00001) and a randomized effect model is used for analysis. The joint tenderness symptom score of the combined group is significantly lower than that of the traditional Chinese medicine fumigation group, and the difference is statistically significant (RR: −0.90, 95% CI: (−0.98, −0.82), *P* < 0.00001).  Figure 9 shows meta-analysis of the joint tenderness symptom score of acupuncture combined with Chinese herbal fumigation in RA. It is clearly evident from Figure 8 that acupuncture combined with traditional Chinese medicine fumigation can alleviate the symptoms of joint tenderness in RA patients.

The article "Investigation of the Clinical Efficacy of Acupuncture Combined with Traditional Chinese Medicine Fumigation in the Treatment of Rheumatoid Arthritis by Meta-Analysis" was retracted in 2023. Reasons: signs of a paper mill; suspected computer-generated content; unreliable results or conclusions; concerns about the data.

## 5. Conclusion

The experimental results show that acupuncture combined with traditional Chinese medicine fumigation can improve the clinical efficacy of RA patients, promote the rapid regression of joint swelling, tenderness, and morning stiffness, and reduce the CRP level of patients, which is worthy of clinical promotion. However, there are still some shortcomings in this study, such as the small scope of literature screening and the small number of literature, which may lead to research results errors and literature heterogeneity. In addition, this study retrieval index only considers the CRP as an inflammatory index, and future research can expand the scope of literature retrieval and retrieval keywords, sufficient sample size, and high quality information data on the basis of meta-analysis to improve the reliability of meta-analysis results.

## Figures and Tables

**Figure 1:** Flowchart of literature screening (Figure 1 is reproduced from Reference [12] (under the Creative Commons Attribution License/public domain)).

**Figure 2:** Overall literature publication bias.

**Figure 3:** Publication bias of single literature.

**Figure 4:** Meta-analysis of therapeutic effects of acupuncture combined with Chinese herbal fumigation on RA.

**Figure 5:** Forest map of CRP meta-analysis of ACUPUNCTURE combined with Chinese herbal fumigation in RA treatment.

**Figure 6:** VAS score meta-analysis of acupuncture combined with Chinese herbal fumigation for RA.

**Figure 7:** Meta-analysis of morning stiffness time of RA treated by acupuncture combined with Chinese herbal fumigation.

**Figure 8:** Meta-analysis of joint swelling symptom score of ACUPUNCTURE combined with Chinese herbal fumigation in RA.

**Figure 9:** Meta-analysis of joint tenderness symptom score of acupuncture combined with Chinese herbal fumigation in RA.

**Table 1:** Basic characteristics of literature.

Author	The year of publication	Outcome index	Quality score
Zhang et al. [13]	2020	ACD	3
Gao [14]	2019	A	2
Qiu and Gao [15]	2020	ACD	4
Pan and Jin [16]	2021	ABEF	5
Gao et al. [17]	2018	AEF	4
Xing [18]	2021	ADE	4
Wu et al. [19]	2020	AEF	4
Wang et al. [20]	2019	AC	3
Guo and Zhou [21]	2019	ACDEF	5
Xu et al. [22]	2021	AC	3
Niu [23]	2015	ACDEF	5
Zhong [24]	2017	A	2
Wang and Zhu [25]	2021	ABDE	5
Zhao [26]	2021	AC	3
Zhou [27]	2019	ACD	4
Chang and Sun [28]	2021	BC	3
Fang et al. [29]	2016	CDEF	5

## Data Availability

The simulation experiment data used to support the findings of this study are available from the corresponding author upon request.
